This article has been retracted.

# The Number of Intraoperative Intestinal Venous Circulating Tumor Cells Is a Prognostic Factor for Colorectal Cancer Patients

**DOI:** 10.1155/2022/4162354

**Published:** 2022-09-23

**Authors:** Zhining Liu, Yimei Gu, Fulong Yu, Lianbang Zhou, Xiaohu Cheng, Heng Jiang, Yang Huang, Yingfeng Zhang, Tongtong Xu, Wenbao Qian, Xianghua Li

**Affiliations:** ^1^Department of General Surgery, The Second Hospital of Anhui Medical University, Hefei, China; ^2^ICU, The First Affiliated Hospital of Anhui Medical University, Hefei, China; ^3^Anhui Medical University, Hefei, China; ^4^Department of Molecular Pathology, Hefei Da'an Medical Laboratory Co., Ltd., Hefei, China; ^5^Guangzhou Da'an Clinical Testing Center Co., Ltd., Guangzhou, China

## Abstract

**Purpose:**

To assess the association between intestinal venous blood (IVB) circulating tumor cells (CTCs) and clinicopathological parameters in stage I-III colorectal cancer (CRC) patients.

**Methods:**

Participants were retrospectively retrieved, who were admitted to our hospital or took annual physical exams between December 1, 2015 and December 31, 2018. A negative enrichment-immunofluorescence in situ hybridization (NE-imFISH) technique was used to isolate and identify CTCs. Receiver operating characteristic (ROC) curves and Youden index values were used to determine the critical CTC cutoff value for the diagnosis of CRC. Kaplan-Meier and log-rank methods were used to conduct survival analyses, and multivariate Cox regression analyses were employed for multivariate corrections to comprehensively evaluate the value of CTCs in the diagnosis of CRC. Relationships between IVB CTCs, clinicopathological parameters, and prognosis were then analyzed based upon patient postoperative follow-up data.

**Results:**

In total, we retrieved 282 patients including 48 healthy controls, 72 patients with benign colorectal tumors, and 162 CRC patients. CRC patients exhibited significantly higher numbers of CTCs relative to control patients or those with benign disease. CTC numbers in CRC patient peripheral blood (PB) and IVB were closely associated with tumor node metastasis (TNM) staging (*P* < 0.01), carbohydrate antigen-125 (CA-125) levels (*P* < 0.001), and KRAS (Kirsten rat sarcoma virus oncogene) mutation status (*P* < 0.001). The disease-free survival (DFS) of patients in the CTC-negative group was significantly longer than that of patients in the CTC-positive group (24.60 ± 13.31 months vs. 18.70 ± 10.19 months, *P* < 0.05), with the same being true with respect to their overall survival (OS) (30.60 ± 12.44 months vs. 35.25 ± 11.57 months, *P* < 0.05). A multivariate analysis revealed that the detection ≥2 CTCs/3.2 ml was independently associated with poorer DFS and OS. CTC counts were independently predictive of CRC patients TNM staging, CA-125, and KRAS mutation status in both univariate and multivariate Cox proportional hazards regression analyses.

**Conclusion:**

CTCs are valuable biomarkers that can be monitored to predict CRC patient disease progression.

## 1. Introduction

Hypoxia has been reported to be associated with poor prognosis and therapeutic resistance in colorectal cancer (CRC) patients. CRC remains the third most prevalent form of cancer globally, [1] and patients are most commonly treated with combination of chemotherapy, radiotherapy, immunotherapy, and radical tumor resection. The overall 5-year survival among CRC patients is reported to range from 50 to 60%, with tumor recurrence and metastasis being the primary drivers of patient mortality [2, 3]. To date, no effective biomarkers have been identified that enable clinicians to readily evaluate disease progression in individual CRC patients in a dynamic fashion. In China, fewer than 15% of CRC patients are diagnosed with this disease while it is still in its early stages. Recent therapeutic advances have prolonged the survival of CRC patients significantly, with 5-fluorouracil (5-FU) or Capecitabine-based chemotherapy administered every 2 (mFOLFOX6) or 3 weeks (CAPEOX) treatments having been associated with marked improvements in CRC-related survival outcomes [4, 5]. However, roughly half of CRC patients present with locally advanced disease or distant metastases upon initial evaluation. It is thus vital that novel strategies for diagnosing and postoperatively monitoring CRC patients be developed in order to improve survival outcomes in these individuals.

While a number of traditional imaging approaches are used to evaluate tumor progression in CRC patients, these modalities have limitations that may fail to fully or accurately reflect disease status in individuals undergoing targeted therapy, chemotherapy, or radiotherapy [6, 7]. Alternatively, a tumor may become necrotic following treatment even though its size appears unchanged, or a tumor may shrink to the point that residual tumor cells are no longer detectable using these imaging approaches. National Comprehensive Cancer Network (NCCN) guidelines for efficacy evaluation do not include tumor markers at present. As such, it remains challenging to accurately identify patients at risk of rapid disease progression. The reliable detection of these high-risk patients would potentially enable clinicians to pursue more aggressive treatment courses in these cases in order to prolong survival and improve quality of life. Circulating tumor cells (CTCs) are cancerous cells that escape from the primary tumor site into circulation, whereupon they have the potential to give rise to distant metastases. Primary tumor-derived CTCs are thought to be the main drivers of tumor metastasis, progression, and chemoresistance. Successful CTC detection has been achieved for most solid tumor types, and CTC counts are correlated with patient prognosis and with the risk of recurrence or metastasis [6, 7]. CTC detection has previously been used to evaluate patients with breast, prostate, thyroid, renal, and colon cancers [8–10]. While CTCs have clear relevance to disease status in individual patients, prior work suggests that only 28.6% of CRC patients exhibits a detectable CTC burden (>1 per 7.5 ml of blood) among Chinese and Western populations [11]. In addition, there is evidence that CTCs are undetectable in the peripheral blood (PB) of patients with stage I-II CRC.

The shedding of tumor cells from the primary tumor into the blood circulation is an early event of cancer metastasis. CRC cells mainly return to the liver through the portal venous system and then enter the artery system to spread through the whole body. CTC counts in the interstitial venous blood (IVB) of CRC patients may be more sensitive than counts in the PB from these same patients, suggesting that IVB samples may be a more reliable target for CRC patient evaluation [11]. Meanwhile, studies have found that the increase of CEA antigen expression in interstitial venous blood is more indicative of postoperative prognosis and the risk of recurrence and metastasis than that of peripheral blood CEA antigen [12]. Intraoperative portal vein blood changes in the expression of miR-497 have higher sensitivity in predicting CRC liver metastasis than in peripheral blood miR-497 and are closely related to the important pathological features, liver metastasis, and prognosis of CRC [13]. As such, in the present study we obtained samples of PB or IVB from healthy controls (PB only), patients with benign tumors (PB only), and CRC patients (both PB and IVB) to evaluate the relationship between CTC counts and patient clinicopathological features and prognosis. Overall, our findings emphasize the value of IVB CTCs as a tool for monitoring CRC disease progression and therapeutic responsiveness.

## 2. Materials and Methods

This study was approved by The Second Hospital of Anhui Medical University Ethics Committee on Medical Research. Informed consents were obtained from the participants.

### 2.1. Sample Collection

CRC patients were diagnosed based upon the 2015 edition of the protocol of diagnosis and treatment of CRC, [14] and the clinical manifestations, disease and family history, physical examination, routine laboratory examinations and molecular tests, endoscopy, imaging, and histopathology were included. Study inclusion criteria were: (1) patients >18 years old. (2) Patients had pathologically confirmed stage I-III CRC, and data were available pertaining to clinicopathological variables including age; sex; tumor diameter; tumor location; tumor histological differentiation; depth of invasion; lymph node metastasis; TNM stage; CTC counts; and AFP, CEA, CA19-9, CA-125, and CA72-4 levels. (3) Available IVB samples had been collected intraoperatively from these patients. (4) Patients provided written informed consent to participate and complied with study follow-up protocols. Study exclusion criteria were (1) patients exhibited evidence of a second primary tumor or (2) patients had previously undergone immunotherapy or radiotherapy treatment or (3) patients had other serious diseases with the potential to impact CRC prognosis.

After treatment, patients underwent physical analyses, liver ultrasound imaging, tumor marker analyses, and other examinations every 3 months. Thoracic and abdominal CT, colonoscopy, and bone scans were performed every 6–12 months. All patients were followed up regularly by telephone, and postoperative follow-up results were collected. Patient death or loss to follow-up was the primary endpoint. In total, 162 patients with CRC were followed, among whom 28 were lost to follow-up, with a follow-up rate of 82.72%. Owing to time constraints, the most recent follow-up date was December 31, 2020, and the longest follow-up time was 5 years and the shortest follow-up time was 2 years. We studied patients followed for at least 3 years. During the follow-up period, there were 51 cases of recurrence and metastasis, including 33 cases of liver metastasis and 18 cases of local recurrence. Overall, 31 patients died during this period, including 27 cases with liver metastases and 4 cases with local recurrence.

The intestinal venous blood was drawn according to the location of the tumor during the operation of CRC tumor resection. In order to minimize the impact of reflux vein influence (splenic vein and other reflux veins) when assessing the relative sensitivity of CTC detection in IVB samples, blood was collected from the first branch vein associated with the primary tumor site as follows: for tumors of the right colon, blood was collected from the superior mesenteric vein (Figure 1(a)). For tumors of the left colon and rectum, blood was collected from the mesenteric lower venous blood supply (Figure 1(b)). We isolated the first reflux vein and conducted a bloodless dissection in an effort to prevent tumor cells or proximal epithelial cells from entering into circulation. We then intraoperatively collected 5 ml of IVB from all patients during CRC tumor resection. The conditions and precautious of IVB sampling was subject to the WHO Guidelines on Drawing Blood. Next, 3.2 ml of these IVB samples were analyzed for CTC counts using a Cyttel® immunofluorescence in situ hybridization (imFISH) approach.

### 2.2. Enrichment and Identification of CRC CTCs

We used 5 ml of IVB from CRC patients in order to enrich CTCs as in prior studies [15]. First, we lysed all red blood cells (RBCs) in IVB samples, after which the remaining cells were suspended in PBS and stained for 30 min with antileukocyte monoclonal antibodies (anti-CD45, Cyttel Biosciences Inc., Jiangsu, China) coated magnetic beads [16]. CD45-positive cells were then magnetically separated, and CRC CTCs were identified via CD45-fluorescence in situ hybridization (FISH) by combining FISH labeling with human chromosome 8 centromere probes (CEP8, orange, Cyttel) and anti-CD45 monoclonal antibodies. Briefly, we began by hybridizing samples with probes specific for CEP8 for 20 min at 37°C, after which samples were washed for 20 min at 43°C in 50% formamide. Next, samples were soaked in 2 × saline sodium citrate (SSC) (Cyttel) at 37°C for 12 min and subjected to gradient alcohol immersion in 75% ethanol for 2 min, 85% for 2 min, and 100% ethanol for 4 min. Samples were washed two times using 20 *μ*l 0.2% bovine serum albumin (BSA) (Cyttel) prior to labeling for 90 min with 180 *μ*l Alexa-Fluor-594- (AF594-) conjugated anti-CD45 (anti-CD45: BSA = 1 : 10). After additional washing with 0.2% BSA, samples were mounted using VECTASHIELD containing DAPI (Cyttel). The sample should be observed entirely along ‘‘S” track [17] with a microscope (Nikon), with CTCs being identified as hyperdiploid cells that were CEP8+/DAPI + /CD45−.

### 2.3. Serum Tumor Marker Analyses

Peripheral blood (3 ml) was collected into anticoagulant-free tubes and centrifuged (1,500 g) at room temperature for 10 min. The AFP, CEA, CA19-9, CA-125, and CA72-4 levels in supernatant serum were determined using an automatic immunoassay analyzer (Cobas e601, Roche, IN, USA). Positive diagnostic criteria for serum tumor markers were defined as levels outside the normal reference range.

### 2.4. DNA Extraction

Tumor DNA was isolated by first having two pathologists independently evaluate H&E-stained 5 *μ*m tumor sections in order to confirm tumor histopathology. Tumor-rich paraffin-embedded sections (>70% tumor tissue) were then selected, and stromal sections were trimmed away using H&E-stained sections for guidance. The remaining tumor tissue was then transferred into a lysis buffer and DNA was isolated based on directions provided with the QIAGEN QIAamp DNA FFPE Tissue Kit (Cat no. 56404, Qiagen, Shanghai, China). A 50 *μ*L volume of ATE buffer was employed for DNA sample elution.

### 2.5. Evaluation of KRAS Mutation Status via Amplification-Refractory Mutation System-Polymerase Chain Reaction (ARMS-PCR)

Mutations in exons 2–4 of the KRAS gene were evaluated with a Chinese-Food-and-Drug-Administration- (CFDA-) approved AmoyDx Human KRAS Mutation Detection Kit (Amoy Diagnostics Co., Ltd., Xiamen, China). DNA quality was assessed via the amplification of an appropriate housekeeping gene and through the use of the HEX channel provided with the kit. A 47-cycle amplification approach was used for this analysis (95°C for 5 min, 1 cycle; 95°C for 25 s, 64°C for 20 s, and 72°C for 20 s, 15 cycles; and 93°C for 25 s, 60°C for 35 s, and 72°C for 20 s, 31 cycles). During the third stage, we collected HEX and FAM signals, with results being interpreted based upon provided instructions.

### 2.6. Statistical Analysis

SPSS v22.0 (SPSS Inc., IL, USA) was used for all statistical testing. Chi-square tests were used for count variables, with risk ratios to assess the prognostic values. Relationships between CTC counts and clinicopathological findings were assessed via logistic regression analyses. Student's *t*-tests were conducted to compare the measurement difference between two groups, and one-way analysis of variance for comparing the difference between multiple groups. The GraphPad Prism (v8.0., CA, USA) was used for figure preparation. Discriminative power was evaluated based upon the area under the ROC curve (AUC), while the optimal CTC cutoff values were selected based upon the Youden Index (sensitivity+1-specificity). A *P* value less than 0.05 (2-sided) was the significance threshold.

## 3. Results

### 3.1. Patient Clinicopathological Findings

Between December 2015 and December 2018, a total of 48 healthy volunteers (25 males and 23 females, with an average age of 45.27 ± 11.73 years) were selected as the blank control group. A total of 72 patients with benign tumors were collected during the same period, including 39 males and 33 females, with an average age of 49.03 ± 13.43 years. We enrolled 162 total CRC patients at the Second Affiliated Hospital of Anhui Medical University. We began by evaluating the clinical characteristics of the 162 CRC patients enrolled in the present study (Table 1). These patients were 33.33% female and 66.67% male (*n* = 54 and *n* = 108, respectively), with a median age of 59.97 ± 13.35 years (range: 26–84). Primary tumors were localized to the rectum, right colon, and left colon in 60, 61, and 41 patients, respectively. With respect to tumor histological differentiation, 51 patients exhibited poorly differentiated tumors, 107 patients exhibited moderately differentiated tumors, and 4 patients exhibited well-differentiated tumors. Tumors were >4 cm and ≤4 cm in 105 and 57 patients, respectively. Tumor invasion depth was graded as T1-T2 in 42 patients and as T3-T4 in 120 patients, while lymph node metastasis was observed in 12 patients. The TNM staging of these CRC patients indicated that 37, 87, and 38 patients had stage I, stage II, and stage III tumors, respectively. Results of IVB tumor marker analyses were as follows: AFP (≤7.00 ng/ml, 110 patients; >7.00 ng/ml, 52 patients), CEA (≤5.20 ng/ml, 91 patients; >5.20 ng/ml, 71 patients), CA19-9 (≤27.00 U/ml, 71 patients; >27.00 U/ml, 91 patients), CA-125 (≤35.00 U/ml, 58 patients; >35.00 U/ml, 104 patients), and CA72-4 (≤6.90 U/ml, 44 patients; >6.90 U/ml, 118 patients).

### 3.2. IVB CTC Cutoff Values in CRC Patients Are More Sensitive than PB CTC Cutoff Values

We enriched for and quantified CTCs in our PB and IVB samples as in prior studies. Briefly, enriched CTCs underwent imFISH staining and anti-CD45/anti-CEP8 staining, with DAPI being used for nuclear staining. CTCs were defined as CEP8+/DAPI+/CD45-cells. We utilized ROC curves to determine the threshold for distinguishing CRC patients from healthy controls. When the cutoff value was set as 1 CTC, 2 CTCs, and 3 CTCs, the AUC and Youden index values were maximal (AUC = 0.9398; Youden index = 0.7778). As such, a CTC count of 2 per 3.2 ml of blood was defined as the diagnostic threshold for CRC, with a corresponding sensitivity of 77.78% and specificity of 100.00% (Figure 2). This was consistent with previous reports [18, 19].

When fewer than 2 CTCs were detected in a given sample, this was considered to be a false positive result. However, greater than or equal to 2 CTCs was considered to be a positive result (Figures 3(a)–3(f)). We found that CTCs isolated from IVB samples exhibited viability comparable to that of cells isolated from whole blood samples (Figure 3(g)). We did not detect any instances of CTC positivity (CTC counts of ≥2 cells per 3.2 ml) in healthy control or benign CRC patients, as expected. In contrast, rates of CTC positivity among CRC patient IVB samples (77.78%) were significantly higher than in PB samples from these same patients (34.57%) (*P* < 0.001; Table 2). These results thus suggest that IVB CTCs are specifically associated with CRC (Figure 4).

### 3.3. CTC Counts Are Positively Correlated with CRC TNM Staging and CA-125 Levels

We next evaluated the relationship between CTC counts and patient clinicopathological findings, revealing these counts to be associated with tumor TNM staging (*P* < 0.001) and CA-125 levels (*P* < 0.001, Table 2 and Figures 5 and 6). An AUC analysis suggested that >3 CTCs were predictive of tumor infiltration and a higher tumor TNM staging (specificity 100.00%, sensitivity 66.05%), while fewer than 3 CTCs were related to *in situ* I staging. We did not detect any association between CTC counts and patient sex, age, tumor diameter, tumor location, tumor histological differentiation, depth of invasion, lymph node metastases, or AFP, CEA, CA19-9, or CA72-4 levels. These results suggest that CTC counts are associated with both tumor TNM staging and CA-125 levels in CRC patients.

### 3.4. The Association between CTCs and KRAS Mutation Status

CRC patients commonly exhibit mutations in exons 2–4 of the KRAS gene [20]. As such, we evaluated KRAS mutation status in the 162 CRC patients in the present study. A total of 74 of these patients (45.68%) harbored KRAS mutations, with 40.74% of patients exhibiting mutations in exon 2, 1.86% of patients exhibiting mutations in exon 3, and 3.09% of patients exhibiting mutations in exon 4 (Table 3). A total of 78.79% of the identified exon 2 KRAS mutations were located within codon 12, whereas 21.21% were within codon 13. The G12D mutation accounted for 32.10% of detected exon 2 mutations. KRAS mutations in CRC patients are associated with resistance to treatment using cetuximab, which is a monoclonal antibody specific for epidermal growth factor receptor (EGFR) [21, 22]. We next assessed the relationship between CTC counts and KRAS mutation (Figure 7) status in DNA samples isolated from FFPE tumor tissue sections (Figure 8). We observed CTC positivity in 64.77% of patients with KRAS-negative CRC, whereas 93.24% of patients exhibiting KRAS mutations were CTC-positive (Table 4; Figure 7; *P* < 0.001). We found that 96.15% of patients exhibiting codon 12 mutations were CTC positive, as were 92.86% of patients with codon 13 mutations, 66.67% of patients with codon 61 mutations, 100.00% of patients with codon 117 mutations, and 66.67% of patients with codon 146 deletions (Table 5). We did not detect any evidence of KRAS mutations in samples from healthy control or benign CRC patients.

### 3.5. The Association between CTC Counts and Patient Prognosis

Kaplan-Meier and log-rank analyses revealed that the median disease-free survival (DFS) of CTC-positive patients was 18.70 months (7.20–35.80 months) and that of CTC-negative patients was 24.60 months (10.80–33.6 months). The median DFS of CTC-positive patients was shorter than that of CTC-negative patients (*P* < 0.05, Figure 9(a)). The median overall survival (OS) of CTC-positive patients was 30.60 months (16.80–35.40 months), while that of CTC-negative patients was 35.25 months (28.80–35.90 months). The median OS of CTC-positive patients was shorter than that of CTC-negative patients (*P* < 0.05, Figure 9(b)).

### 3.6. Univariate and Multivariate Analyses of CRC Patient Prognosis

A univariate Cox proportional risk regression model was used to analyze the relationships between prognosis and age, sex, tumor location, tumor diameter, tumor histological differentiation, invasion depth, lymph node metastasis, TNM staging, AFP, CEA, CA19-9, CA72-4, or CA-125 levels, KRAS mutation status, and CTC counts. The degree of tumor differentiation, lymph node metastasis, TNM staging, CA125 > 35.00 U/ml, KRAS mutations, and CTC counts ≥2 per 3.2 ml were significantly associated with DFS (*P* < 0.05, Table 6). The degree of tumor tissue invasion, TNM staging, KRAS mutation, and CTC counts ≥2 per 3.2 ml were also significantly associated with shorter OS (*P* < 0.05, Table 6). A multivariate Cox proportional risk regression model analysis revealed that CTC counts ≥2 per 3.2 ml and KRAS mutation status were independent predictors of DFS (*P* < 0.05, Table 7), while CTC counts ≥2 per 3.2 ml, KRAS mutation status, TNM staging, and CA-125 levels >35.00 U/ml were independent predictors of OS (*P* < 0.05, Table 8).

## 4. Discussion

There have been many recent advances in the field of CRC treatment, with numerous efforts made to establish strategies for diagnosing and treating CRC in a manner that prevents tumor recurrence or metastatic progression. Metastasis is a primary cause of death among CRC patients, [23] and detecting such metastasis at an early stage is essential for improving therapeutic responsiveness [24]. Even when CRC is detected at an early stage; however, it often recurs postoperatively within a 5-year period [25]. CTC detection has been explored as a relatively noninvasive means of monitoring and diagnosing CRC patients [26]. CTCs are released into circulation from primary tumors, and previous research has identified a direct relationship between CTC shedding and clinical CRC patient outcomes such as metastasis, recurrence, and therapeutic responsiveness. At present, however, approaches to detecting CTCs in CRC patients are hampered by their relatively low sensitivity and specificity.

The high sensitivity of IVB samples for the detection of CTCs may be attributable to two factors. First, CTCs from the primary tumor site are released into the intestinal vein, resulting in a higher local CTC concentration in the IVB [27]. Second, the liver is the only organ that can block IVB flow into the peripheral veins and can thus act as a filter to regulate the release of CTCs into the periphery [28]. We identified CRCs by first enriching for CD45-negative cells prior to staining for CD45 and CEP8 with appropriate antibodies and probes, as this approach has been shown to be highly sensitive and specific [17, 29]. We analyzed data pertaining to 162 CRC patients, of whom 77.78% were found to exhibit CTC enrichment, suggesting that such enrichment is a sensitive marker of CRC. Such CTCs may thus be a valuable diagnostic or prognostic biomarker in patients with malignant CRC [6].

We found that CTC counts in CRC patients were significantly associated with both CA-125 and with TNM staging, consistent with prior findings [11]. These results suggested that CTCs are associated with tumor progression, metastasis, and tumor marker screening, in line with prior work [11]. While traditional imaging approaches are of limited utility when evaluating the risk of distant metastasis in patients with stage I disease without lymph node metastases, we found that CTC counts were more sensitive than such imaging approaches. Further research will be needed to establish more sensitive approaches to detecting CTCs in patients in which the cells are not highly abundant, and it is also essential that identified CTCs be assessed in order to ensure that they are derived from the primary tumor site.

The KRAS gene is among the most commonly mutated genes in many human cancers, given that it functions as a key intracellular regulator of cell growth signaling. Dysregulated or mutated KRAS can cause erroneous growth of cells when they should not, resulting in uncontrolled cell proliferation and oncogenesis [30, 31]. In line with previous studies [19], we found that the most prevalent mutation was KRAS G12D, followed by the G12V, G13D, G12S, G12A, G12C, G12R, and G13C mutations. KRAS mutation status is associated with cetuximab resistance in CRC patients, and as such, it is important that KRAS mutation status be assessed in patients prior to cetuximab administration [32]. Cetuximab is efficacious in CRC patients with wild type (WT) KRAS and exhibits some reduced efficacy in patients bearing the G13D mutation [33]. Our results showed the diagnostic and prognostic utility of CTC counts in individuals suffering from CRC.

In the present study, we utilized a CD45-negative enrichment and CEP8-FISH strategy in order to detect CTCs with a higher degree of sensitivity [28]. Herein, we found that this CEP8-CD45-FISH-based strategy yielded higher sensitivity than did the detection of the tumor markers AFP, CEA, CA19-9, and CA72-4. However, CTC sensitivity was similar to that of the tumor marker CA-125. These results thus suggest that CTCs may be of moderate utility as a tool for CRC diagnosis. Despite their apparent value, future research will be essential in order to develop optimized approaches to isolating CTCs with higher sensitivity and specificity rates. Such strategies may rely upon the use of chromosome enumeration probes or on staining for tumor-specific antigens in order to more accurately detect CTCs.

In this study, we found that CTC counts were correlated with patient prognosis. The presence of ≥2 CTCs per 3.2 ml of blood and KRAS mutations were independent adverse prognostic factors associated with DFS, while TNM staging, CA-125 levels, CTCs ≥2 per 3.2 ml, and KRAS mutations were independent adverse prognostic factors associated with OS, consistent with the results of Yang et al. [34] who analyzed 211 cases of stage I-III CRC and similarly identified intraoperative CTC positivity as an independent indicator of poor prognosis. Patients exhibiting intraoperative CTC positivity had a higher risk of recurrence relative to patients exhibiting intraoperative CTC-negativity. Therefore, intraoperative CTC detection is of key clinical significance, as it can independently predict the progression and survival of CRC patients, enabling appropriate patient treatment planning to facilitate more efficacious individualized treatment.

There are certain limitations to this analysis. For one, our sample size was limited, and as such, future large-scale studies will be needed to validate these findings. Additional studies will also be required to assess the diagnostic or prognostic utility of CTCs in combination with other biomarkers or readouts in CRC patients in order to better understand their association with patient treatment and clinical outcomes. Future large-scale multicenter studies will be invaluable as a means of assessing the prognostic relevance of CTCs in CRC patients, thus laying the foundation for personalized CRC treatment in affected patients. Other parameters could also be investigated [35–38].

## 5. Conclusion

In summary, our results indicate that CTCs counts in CRC patients are associated with CA-125 levels, TNM staging, and KRAS mutation status. A such, CTCs may represent a valuable biomarker that can be used to monitor CRC progression in patients.

## Figures and Tables

**Figure 1:** The collection of intestinal venous blood from different patient tumor sites. (a) For tumors of the right colon, blood was collected from the superior mesenteric vein. (b) For tumors of the left colon and the rectum, blood was collected from the mesenteric lower venous blood supply.

**Figure 2:** The sensitivity of CTCs for the diagnosis of colorectal cancer was compared using a receiver operating curve analysis. GraphPad Prism (v8.0. CA, USA) was used for figure construction, *P* < 0.001.

**Figure 3:** Immunostaining profiles of CTCs isolated from the IVB of CRC patients. CTCs from these patients underwent imFISH staining, with CTCs being identified as cells staining positive for anti-human CEP8, but negative for antihuman CD45. (a) Positive control group. (b) CTC = 0. (c) CTC = 22. (d) CTC = 12. (e) CTC = 6. (f) CTC = 1. Identified CTCs exhibited normal morphological findings upon microscopic evaluation (400x). As per the above Figures 3(a)–3(f), space is limited, not showing all the results. (g) The mean viability of enriched tumor cells (yellow) and WBCs (red) was 98.67 ± 0.88% and 95.20 ± 1.38% (mean ± SD), respectively. Data are representative images of three independent experiments. Asterisks were marked to show the significance of tumor cells group compared with WBCs group (^*∗∗∗*^*P* < 0.001). CTCs, circulating tumor cells; imFISH, immunofluorescence in situ hybridization; CD45, leukocyte-specific antibodies; CEP8, human chromosome 8 specific sequence; DAPI, 4′,6-diamidino-2-phenylindole; MERGE, CD45 + CEP8 + DAPI; WBCs, whole blood cells.

**Figure 4:** CTC counts distributions in CRC patient IVB (*n* = 162, range, 0–22), CRC patient PB (*n* = 162, range, 0–6), benign CRC patient PB (*n* = 72, range, 0-1), and healthy controls (*n* = 48, range, 0-1). GraphPad Prism (v8.0. CA, USA) was used for figure construction, ^*∗∗∗*^*P* < 0.001, ns, *P* > 0.05. CTCs, circulating tumor cells.

**Figure 5:** CTC counts distributions in CRC patients as a function of pathological stage. GraphPad Prism (v8.0. CA, USA) was used for figure construction, ^*∗∗∗*^*P* < 0.001, ^*∗∗*^*P* < 0.01, ns, *P* > 0.05. CTCs, circulating tumor cells.

**Figure 6:** CTC counts distributions in CRC patients as a function of CA-125. GraphPad Prism (v8.0. CA, USA) was used for figure construction, ^*∗∗∗*^*P* < 0.001. CTCs, circulating tumor cells.

**Figure 7:** CTC counts distributions in CRC mutation of KRAS. GraphPad Prism (v8.0. CA, USA) was used for figure construction, ^*∗∗∗*^*P* < 0.001. CTCs, circulating tumor cells.

**Figure 8:** KRAS gene mutations in four exons [2, 3, 4] and codons [12, 13, 61, 117, 146]. (a) A codon 12 mutation in exon 2 of patient CRC-3. (b) A codon 13 mutation in exon 2 of patient CRC-35. (c) A codon 61 mutation in exon 3 of patient CRC-81. (d) A codon 117 mutation detected in exon 4 of patient CRC-114. (e) A codon 146 mutation detected in exon 4 of patient CRC-150. (f) No mutations were detected in three exons in patient CRC-2. These findings are representative of our findings among the 162 CRC patients in this study.

**Figure 9:** The relationship between CTC counts before and during surgery, disease-free survival, and overall survival. (a) Among 51 patients with CRC, the median DFS in CTC-positive patients was shorter than in CTC-negative patients, *P* < 0.05. (b) Among 33 CRC patients, the median OS of CTC-positive patients was shorter than that of CTC-negative patients, *P* < 0.05.

**Table 1:** The association between IVB CTC counts and patient clinicopathological findings.

Variations	*N*	Positive/negative	CTCs-positive (%)	*χ* ^2^	*P*-value
Gender				1.446	0.229
Male	108	87/21	80.56		
Female	54	39/15	72.22		

Age/years				0.177	0.674
≤60	77	61/16	79.22		
>60	85	65/20	76.47		

Tumor location				0.604	0.739
Left colon	41	32/9	78.04		
Right colon	61	37/14	52.46		
Rectum	60	47/13	78.33		

Histologic differentiated				1.990	0.370
Poorly	51	41/10	80.39		
Moderately	107	83/24	77.57		
Well	4	2/2	50.00		

Diameter/cm				2.105	0.147
≤4.0	57	48/9	84.21		
>4.0	105	78/27	74.29		

Invasion depth				2.066	0.151
T1-T2	42	36/6	85.71		
T3-T4	120	90/30	75.00		

Lymph node metastasis				0.231	0.630
Negative	150	116/34	77.33		
Positive	12	10/2	83.33		

TNM staging				12.091	0.002
I	37	31/6	83.78		
II	87	59/28	67.82		
III	38	36/2	94.74		

AFP (ng/ml)				1.070	0.301
≤7.0	110	83/27	75.45		
>7.0	52	43/9	82.69		

CEA (ng/ml)				0.458	0.498
≤5.2	91	69/22	75.82		
>5.2	71	57/14	80.28		

CA19-9 (U/ml)				0.007	0.933
≤27	71	55/16	77.46		
>27	91	71/20	78.02		

CA-125 (U/ml)				50.968	0.000
≤35	58	27/31	46.55		
>35	104	99/5	95.19		
>35	104	99/5	95.19		
CA72-4 (U/ml)				0.270	0.604
≤6.9	44	33/11	75.00		
>6.9	118	93/25	78.81		

CTCs, circulating tumor cells; AFP, alpha-fetoprotein; CEA, carcinoembryonic antigen; CA19-9, glycoprotein antigen 199; CA-125, glycoprotein antigen 125; CA72-4, glycoprotein antigen 72-4.

**Table 2:** Differences in CTC detection among healthy control, benign CRC, and CRC patient groups.

Variable	Collecting blood position	*n*	Positive/negative	CTCs-positive (%)	*χ* ^2^	*P*-value
Healthy controls	Peripheral venous blood	48	0/48	0	176.756	0.000
Benign CRC	Peripheral venous blood	72	0/72	0		
CRC	Peripheral venous blood	162	56/106	34.57		
CRC	Intestinal venous blood	162	126/36	77.78		

CTCs, circulating tumor cells; CRC, colorectal cancer.

**Table 3:** KRAS mutation types detected among 162 CRC patients.

Gene	Exon	Codon	Mutation	Numbers of mutations (% of 162)
KRAS	2	12, 13	G12S, G12D, G12C, G12R, G12V, G12A, G13C, G13D	66 (40.74%)
	3	61	Q61L, Q61R, Q61H	3 (1.86%)
	4	117, 146	K117N, A146T, A146V, A146P	5 (3.09%)

KRAS, Kirsten rat sarcoma virus oncogene.

**Table 4:** The association between CTC counts and KRAS mutation status.

Variable	*n*	Positive/negative	CTCs-positive (%)	*χ* ^2^	*P*-value
KRAS	162			18.852	0.000
Mutant type	74	69/5	93.24		
Wild type	88	57/31	64.77		

CTCs, circulating tumor cells; KRAS, Kirsten rat sarcoma virus oncogene.

**Table 5:** The association between CTC counts and KRAS mutation status.

KRAS mutation	*n*	*n*, CTCs-Positive (%)	N, CTCs-Negative (%)
Code12	52	50 (96.15%)	2 (3.85%)
Code13	14	13 (92.86%)	1 (7.14%)
Code61	3	2 (66.67%)	1 (33.33%)
Code117	2	2 (100.00%)	0
Code146	3	2 (66.67%)	1 (33.33%)

CTCs, circulating tumor cells; KRAS, the Kirsten rat sarcoma.

**Table 6:** Univariate analysis of DFS and OS in patients with CRC.

Variations	Univariate analysis (DFS)			Univariate analysis (OS)		
	95% CI	*χ*2	*P*-value	95% CI	*χ*2	*P*-value
Gender	[17.123, 22.077]	0.260	0.610	[17.123, 22.077]	1.227	0.268
Age/years	[18.274, 20.926]	0.002	0.883	[0.000, 50.190]	0.203	0.652
Tumor location	[19.216, 19.984]	1.149	0.563	[15.206, 31.994]	0.954	0.621
Histologic differentiated	[17.458, 21.742]	11.470	0.003	—	0.149	0.928
Diameter/cm	[18.117, 21.023]	0.017	0.897	[12.513, 19.123]	1.118	0.290
Invasion depth	[18.266, 20.934]	0.783	0.376	[13.284, 19.682]	8.475	0.004
Lymph node metastasis	[17.707, 21.493]	12.617	0.000	[14.552, 22.025]	1.707	0.191
TNM staging	[18.660, 20.540]	27.365	0.000	[14.846, 20.391]	12.555	0.002
AFP/(ng/ml)	[18.154, 21.046]	2.789	0.095	[14.243, 21.465]	0.031	0.861
CEA/(ng/ml)	[18.052, 21.148]	1.640	0.200	[13.235, 20.134]	0.720	0.396
CA19-9/(U/ml)	[18.219, 20.981]	0.028	0.867	[13.894, 20.490]	0.849	0.357
CA72-4/(U/ml)	[18.451, 20.749]	0.012	0.914	[14.354, 20.712]	1.066	0.302
CA-125 (U/ml)	[19.237, 19.963]	6.316	0.012	[15.573, 22.109]	3.289	0.070
CTCs	[18.450, 20.750]	5.069	0.024	[19.520, 31.690]	6.992	0.008
KRAS	[17.987, 20.413]	26.139	0.000	[16.672, 23.114]	3.909	0.048

CTCs, circulating tumor cells; AFP, alpha-fetoprotein; CEA, carcinoembryonic antigen; CA19-9, glycoprotein antigen 199; CA-125, glycoprotein antigen 125; CA72-4, glycoprotein antigen 72-4; KRAS, Kirsten rat sarcoma virus oncogene.

**Table 7:** Multivariate analysis of DFS in patients with CRC.

Variable	*β*	SE	Wald *χ*2	Exp (*B*)	95% CI	*P*-value
Gender	0.417	0.710	0.346	1.518	[0.378, 6.098]	0.556
Age/years	0.290	0.553	0.274	1.336	[0.452, 3.946]	0.600
Tumor location	0.629	0.773	0.662	1.876	[0.412, 8.539]	0.416
Histologic differentiated	−2.949	1.665	3.136	0.052	[0.002, 1.370]	0.077
Diameter/cm	−0.446	0.544	0.735	0.627	[0.216, 1.821]	0.391
Invasion depth	−0.302	0.835	0.131	0.739	[0.144, 3.798]	0.718
Lymph node metastasis	−0.631	0.763	0.683	0.532	[0.119, 2.376]	0.409
TNM staging	1.403	0.952	2.172	4.068	[0.629, 26.299]	0.141
AFP/(ng/ml)	0.494	0.581	0.723	1.638	[0.525, 5.112]	0.395
CEA/(ng/ml)	0.464	0.749	0.384	1.590	[0.367, 6.901]	0.536
CA19-9/(U/ml)	0.618	0.687	0.810	1.855	[0.483, 7.128]	0.368
CA72-4/(U/ml)	0.487	0.675	0.520	1.628	[0.433, 6.116]	0.471
CA-125 (U/ml)	0.022	0.699	0.001	1.022	[0260, 4.020]	0.975
CTCs (n/3.2 ml)	1.970	0.974	4.086	7.168	[1.062, 48.391]	0.043
KRAS	1.793	0.814	4.846	6.005	[1.217, 29.623]	0.028

CTCs, circulating tumor cells; AFP, alpha-fetoprotein; CEA, carcinoembryonic antigen; CA19-9, glycoprotein antigen 199; CA-125, glycoprotein antigen 125; CA72-4, glycoprotein antigen 72-4; KRAS, Kirsten rat sarcoma virus oncogene.

**Table 8:** Multivariate analysis of OS in patients with CRC.

Variable	*β*	Se	Wald *χ*2	Exp (*B*)	95% CI	*P-*value
Gender	0.995	0.621	2.369	2.599	[0.770, 8.774]	0.124
Age/years	−1.122	0.776	2.090	0.326	[0.071, 1.491]	0.148
Tumor location	0.129	1.014	0.016	1.137	[0.156, 8.300]	0.899
Histologic differentiated	−1.097	0.685	2.564	0.334	[0.087, 1.279]	0.109
Diameter/cm	−0.557	0.845	0.434	0.573	[0.109, 3.004]	0.510
Invasion depth	−2.113	1.259	2.818	0.121	[0.010, 1.425]	0.093
Lymph node metastasis	0.219	1.017	0.047	1.245	[0.170, 9.135]	0.829
TNM staging	2.553	1.140	5.015	12.847	[1.375, 119.998]	0.025
AFP/(ng/ml)	−1.233	0.857	2.069	0.292	[0.054, 1.564]	0.150
CEA/(ng/ml)	1.577	1.062	2.205	4.841	[0.604, 38.818]	0.138
CA19-9/(U/ml)	1.375	0.894	2.364	3.956	[0.685, 22.837]	0.124
CA72-4/(U/ml)	−0.984	1.058	0.865	0.374	[0.047, 2.973]	0.352
CA-125 (U/ml)	−3.365	1.307	6.630	0.035	[0.003, 0.448]	0.010
CTCs (n/3.2 ml)	−3.813	1.239	9.467	0.022	[0.002, 0.251]	0.001
KRAS	2.235	0.880	6.447	9.346	[1.665, 52.459]	0.011

CTCs, circulating tumor cells; AFP, alpha-fetoprotein; CEA, carcinoembryonic antigen; CA19-9, glycoprotein antigen 199; CA-125, glycoprotein antigen 125; CA72-4, glycoprotein antigen 72-4; KRAS, Kirsten rat sarcoma virus oncogene.

## Data Availability

The data used to support the findings of this study can be obtained from the corresponding author upon request.
